The article "Adsorption and sensor performance of transition metal-decorated zirconium-doped silicon carbide nanotubes for NO2 gas application: a computational insight" was retracted in 2025. Reasons: errors in the data; errors in the text; original data or images not available; unreliable data.

# Adsorption and sensor performance of transition metal-decorated zirconium-doped silicon carbide nanotubes for NO_2_ gas application: a computational insight†

**DOI:** 10.1039/d3ra08796d

**Published:** 2024-02-12

**Authors:** Ismail O. Amodu, Faith A. Olaojotule, Miracle N. Ogbogu, Oluwatobi A. Olaiya, Innocent Benjamin, Adedapo S. Adeyinka, Hitler Louis

**Affiliations:** a Computational and Bio-Simulation Research Group, University of Calabar Calabar Nigeria louismuzong@gmail.com; b Department of Mathematics, University of Calabar Calabar Nigeria; c Department of Research Analytics, Saveetha Dental College and Hospitals, Saveetha Institute of Medical and Technical Sciences, Saveetha University Chennai India; d Department of Chemical Sciences, University of Johannesburg Pretoria South Africa; e School of Chemistry, University of Leeds Leeds LS2 9JT UK

## Abstract

Owing to the fact that the detection limit of already existing sensor-devices is below 100% efficiency, the use of 3D nanomaterials as detectors and sensors for various pollutants has attracted interest from researchers in this field. Therefore, the sensing potentials of bare and the impact of Cu-group transition metal (Cu, Ag, Au)-functionalized silicon carbide nanotube (SiCNT) nanostructured surfaces were examined towards the efficient detection of NO_2_ gas in the atmosphere. All computational calculations were carried out using the density functional theory (DFT) electronic structure method at the B3LYP-D3(BJ)/def2svp level of theory. The mechanistic results showed that the Cu-functionalized silicon carbide nanotube surface possesses the greatest adsorption energies of −3.780 and −2.925 eV, corresponding to the adsorption at the o-site and n-site, respectively. Furthermore, the lowest energy gap of 2.095 eV for the Cu-functionalized surface indicates that adsorption at the o-site is the most stable. The stability of both adsorption sites on the Cu-functionalized surface was attributed to the small ellipticity (*ε*) values obtained. Sensor mechanisms confirmed that among the surfaces, the Cu-functionalized surface exhibited the best sensing properties, including sensitivity, conductivity, and enhanced adsorption capacity. Hence, the Cu-functionalized SiCNT can be considered a promising choice as a gas sensor material.

## Abstract 2

Owing to the fact that the detection limit of already existing sensor-devices is below 100% efficiency, the use of 3D nanomaterials as detectors and sensors for various pollutants has attracted interest from researchers in this field.

## 1 Introduction

Prevalent diseases such as cancer and stroke account for about a million deaths every year due to the inhalation of microscopic pollutants, which can enter the respiratory and circulatory tracts, causing severe damage to major organs and glands.^1,2^ In 2018, the World Health Organization (WHO) reported that air pollution is one of the major risks to health.^3^ Pollutants are chemical or biological substances that disintegrate the quality of useful resources when introduced in the environment and are known to pose a significant risk to public health.^4^ Nitrogen oxides, a group of highly reactive gases such as nitrogen oxide (NO) and nitrogen dioxide (NO_2_), serve as major contributors to the depleting air quality.^5^ Many anthropogenic activities such as the combustion of fossil fuels significantly contributes to the presence of toxic forms of NO gases and exposure to an enormous amount of NO_2_ has a severe effect on wildlife and humans.^6,7^ Alternatively, a trace amount of NO_2_ is suitable as a fingerprint for tracking chronic obstructive pulmonary disease (COPD).^8^ Nitrogen dioxide (NO_2_) is also a major contributor to the formation of acid rain and photochemical smog and is the major component in the formation of fine particles. It is a primary air pollutant, which also affects the tropospheric ozone.^9^ Human activities including oil spillage, explosives, burning, refining of petrol, and manufacturing of food and natural sources such as volcanoes, oceans, and forest fires significantly contribute to the increasing NO_2_ level. This has caused numerous health problems, especially, respiratory issues such as swelling of the tissues in the throat, reduced oxygenation, and rapid burning, which occur when the lining of the lungs gets inflamed and often triggered by these activities due to the generation of high concentrations of NO_2_ gas molecules.^10,11^

Nanotechnology is the science and technology of creating nanoparticles and manufacturing materials with sizes less than 100 nm.^12^ It incorporates different fields such as physics, chemistry, materials science, and biology to develop the production of biomedical products, high-performance products, and consumer articles.^13^ For example, drug carriers and electrochemical sensors were developed in previous studies using different nanomaterial such as carbon nanotubes and inorganic metal oxides, providing versatile compositions.^14,15^ Additionally, it aids the engineering of the physical properties ranging from the size, morphology, and surface characteristics to the structure of atoms.^16–18^ Heightened therapeutic efficiency and enhanced clinical benefits in surviving cancer have been achieved using nanomedicines such as Doxil for the treatment of sarcomas, which increases the stability and solubility of drugs.^19^ Nano-composite materials are significantly known to include a wide variety of systems including one-dimensional, three-dimensional and amorphous materials.^20–22^ Nanocages are cage-like assemblies of proteins, having three engineerable surfaces, which can be used as potential carriers of molecules for therapeutic and diagnostic purposes.^23,24^ These nanomaterials in form of cages, tubes, and wires also facilitate the safer transportation, delivery, trapping and sensing of different molecules and minimize the premature degradation or interactions of doped atoms in the biological or physical environment.^25–27^

In-depth studies on metal oxide-based NO_2_ sensors have been done by researchers in the past. The active sites on metal oxides are responsible for their sensing characteristics. This implies that the sensing mechanism of different gases depends on the crystallinity and number of defects present in metal oxide-like nanoparticles. Also, these nanostructures can be used for the fabrication of NO_2_ gas sensors due to their specific attributes such as high thermal stability, non-toxicity and high chemical sensitivity.^28–30^ Resistive gas sensors are employed for the detection of variations and concentrations of different ambient gases. In this case, the active layer is the main part of a sensor, which can be composed of various materials including inorganic, organic and hybrid materials.^31,32^ However, the major disadvantages of resistive gas sensors are their limited sensitivity and poor selectivity. Thus, several strategies have been introduced to overcome these shortcomings, including varying the operating temperature of the sensor.^33,34^ In recent studies, Cheng *et al.* reported that gas sensors based on hybrid 1D/3D-structured perovskite provide a new pathway for the highly sensitive and stable detection of NO_2_ gas.^35^ Nwagu *et al.*^36^ reported that K, Ca, Mg and late transition metal dopants enhance the adsorption of SO_2_, which is attributed to the improvement in surface properties. In another study, Inah *et al.* revealed that GQD_N and GQD-S are good adsorbents for the adsorption of C_2_H_4_, CH_4_, and H_2_ gases that exhibit non-covalent interactions, indicating the weak intermolecular interactions between the surface of the adsorbents and gas molecules.^37^

Therefore, the present work focused on adopting more effective and reliable methods for the detection of NO_2_ gas molecules in different sectors ranging from automobiles and industrial plants to farming. Recently, the process of measuring the air quality has been considered to be unaffordable due to the high cost of laboratory equipment and large monitoring devices, which also requires professional operators. Accordingly, the development of alternative devices, procedures and equipment with relatively small size, low cost and promising performances in terms of sensitivity, fast response and low energy consumption will have a positive impact on curbing various pollutants especially NO_2_ gases. Hence, systems with high miniaturization, low cost, and simple production techniques will be of significant interest because the improvement in nanotechnology using engineered nanoparticles has resulted in exceptional efficacy in the biomedical field and designing future sensor devices.

Herein, the current investigation endeavored to provide new insight into the sensing potential of bare and Cu-group transition metal (Cu, Ag, Au)-functionalized silicon carbide nanotube (SiCNT) nanostructured surfaces through a comprehensive computational study. The aim of this investigation was twofold, *i.e.*, to design advanced sensor materials capable of detecting NO_2_ gas molecules with intriguing sensitivity and obtaining detailed knowledge on the nature of the interactions and the stabilization of these materials, which are essential for their gas adsorption mechanisms. Initially, we performed structural optimization to uncover the most stable geometric configurations and the structural properties of the materials under investigation. Furthermore, to probe the sensing properties of the materials, various analyses such as adsorption energy, frontier molecular orbital (FMO), stabilization energy, density of states (DOS), atoms-in-molecules (AIM), reduced density gradient (RDG), molecular dynamic (MD) simulations, and sensor mechanisms were thoroughly performed.

## 2 Computational details

All theoretical calculations were performed using Kohn–Sham (KS) density functional theory (DFT) computation. To obtain the most stable geometric structures, ground-state geometric optimization was carried out for all the structures using the B3LYP-D3(BJ)/def2svp level of theory.^38^ Gaussian 16,^39^ together with its Gauss View 6.0.16 (ref. 40) software graphical interphase was used for sketching, optimization and extraction. Insight into the nature of the interactions, electronic properties, and adsorption energy were gained using the visual study, quantum descriptors, and adsorption energy calculations. The visual study, employing the quantum theory of atoms-in-molecules (QTAIM), and its visual extension, which is the non-covalent interaction (NCI) analysis, were carried out using the Multiwfn 3.7 program,^41^ where the visualization of NCI was done using the visual molecular dynamics (VMD) software.^42^ Also, the density of states (DOS) was computed using the Multiwfn 3.7 program, and subsequently the generated data was plotted using the Origin software. Upon adsorption, the adsorption energy of the resulting complexes was determined using eqn (1), as follows:

1 *E*_ad_ = *E*_Complex_ − (*E*_Surface_ + *E*_Molecule_)

where *E*_Complex_ is the total energy of the resulting complex due to adsorption and *E*_Surface_ denotes the energy of the isolated bare and functionalized SiCNT surfaces. *E*_Molecule_ denotes the energy of the NO_2_ gas molecule and *E*_ad_ denotes the adsorption energy of the resulting complexes. The extraction of the HOMO and LUMO energies was carried out using the Gaussian 16 software and HOMO–LUMO plots from ChemCraft 1.6 program.^43^ In the NVE ensemble, a constant value of particles, energy, and volume with the fixed temperature of 298.00 K were maintained in the molecular dynamic simulations. In all cases, a simulation duration of 10 ps, with a time-step of 1000 steps was employed. The initial condition was randomized, with an assignment of random initial velocities and use of random number seeds, which was approx. 1.6 × 10^8^. This enabled the simulations to be reproduced.

## 3 Results and discussion

### 3.1 Optimizations and molecular geometry

Initially, the geometries of the molecular structures were equilibrated, and the energy minimization was carried out to ensure the stability and sensitivity of the studied systems.^44^ The importance of optimization in the calculation of adsorption energies cannot be overstated, given that it facilitates the calculation of the adsorption energies of the systems of interest. Initially, the silicon carbide nanotube was doped with zirconium, and then further functionalized with transition metals (Cu, Ag, and Au). The surfaces were optimized separately as well as the NO_2_ gas molecule, before being placed together, and then optimized again to form complexes. The morphology of the surfaces was reengineered to obtain a new surface with enhanced functionalities towards sensing. The bond length of the optimized NO_2_ gas molecule was computed, as presented in Fig. 1.

**Fig. 1:** Optimized structure of the NO_2_ gas molecule together with its bond lengths and angle.

Easy glance into the molecular geometries of the structures was possible, as shown in Fig. 1, where the bond lengths between two atoms are shown. Clearly, the bond lengths between two atoms in the NO_2_ gas molecule and that within the rings of the functionalized SiCNT surfaces were visualized. Considering the NO_2_ gas molecule, the bond lengths for the N–O bonds were determined to be 1.192 and 1.192 Å, which were found to be consistent with previous computational studies with a bond length of 1.21 and 1.16 Å in ref. 45 and 46. Also, before functionalizing the surface of SiCNT, the carbon–zirconium bond lengths were computed and found to be 2.082, 2.088, and 2.105 Å for the C_32_–Zr_100_, C_34_–Zr_100_ and C_39_–Zr_100_ bonds, respectively. Similarly, computed the bond lengths are consistent with previous theoretically calculated bond lengths.^47^

Given that the selectivity of a material used as a sensor device is dependent on its properties, it is necessary to enhance the sensing performance of nanomaterials. Thus, the nanotube surface was reengineered with transition metals such as Ag, Au, and Cu, thereby resulting in the formation of Ag_Zr@SiCNT, Au_Zr@SiCNT, and Cu_Zr@SiCNT surfaces respectively. The functionalization was achieved by adding each transition metal to the carbon atom of the already doped Zr@SiCNT surface, as shown in Fig. 2. Also, Fig. 3 presents the optimized structures of the complexes formed as a result of adsorption.

**Fig. 2:** Optimized structures of the bare and functionalized SiCNT surfaces.

**Fig. 3:** Optimized structures of the resulting complexes due to adsorption.

The bond lengths between carbon and zirconium (C–Zr) and that of carbon and silver (C–Ag) were computed before and after adsorption for all the surfaces to gain insight into the effect of adsorption on the morphology of the tubes. This was to determine whether adsorption stretches or shortens the bond lengths. Furthermore, the adsorption distance was computed, which was observed to be between the n-site or o-site of adsorption and transition metals for the functionalized surfaces and between zirconium for the Zr@SiCNT surface. The sites of adsorption were also considered to obtain the best adsorption configurations. The results of the structural geometries are summarized in Table 1. The bond lengths observed for the Z1-X complexes (X = n and o sites) were found to be slightly elongated as a result of adsorption, leading to stretching in the nanotube. For example, the C_32_–Zr_100_ bond increased from 2.082 to 2.119 and 2.217 Å, corresponding to the n-site and o-site of adsorption, respectively. However, the functionalized surfaces exhibited different behavior in their structures. For example, adsorption on the A1-X complexes (X = n and o sites) showed a slight or no effect on their bond lengths, with the same bond length values of 2.083 and 2.089 Å before and after adsorption, and then a slight change from 2.103 to 2.101 and 2.100 Å for the n-site and o-site of adsorption respectively. In the labelled A2-X and C1-X complexes, slight changes were observed in the n-site and o-site of adsorption, depicting that adsorption led to an almost insignificant shift in their geometric structures. Overall, the observed changes in the bond lengths indicate that a reaction occurred, thus establishing the adsorption process. In most cases, a shorter bond length suggests a weak interaction between the adsorbate and adsorbent.^48^ The shortest interaction distances of 1.920 and 1.916 Å, corresponding to the n-site and o-site of adsorption, were found in the Cu-functionalized surfaces, indicating the weakest interactions among the studied surfaces. Alternatively, the strongest interactions were observed in the complex corresponding to the Zr@SiCNT surface, which was not functionalized.

**Table 1:** The computed bond lengths before and after adsorption calculated at the B3LYP-D3(BJ)def2svp level of theory^a^

System	Bond label	Bond length (Å)		
		Before ads.	After ads.	
			n-site	o-site
NO_2__X_Zr@SiCNT (Z1-X)	Q–Zr_100_	—	2.214	2.268
	C_32_–Zr_100_	2.082	2.119	2.217
	C_34_–Zr_100_	2.088	2.120	2.113
	C_39_–Zr_100_	2.105	2.213	2.132
NO_2__X_Ag_Zr@SiCNT (A1-X)	Q–Ag_101_	—	2.118	2.205
	C_23_–Ag_101_	2.629	2.197	2.204
	C_32_–Zr_100_	2.083	2.083	2.083
	C_34_–Zr_100_	2.089	2.089	2.089
	C_39_–Zr_100_	2.103	2.101	2.100
NO_2__X_Au_Zr@SiCNT (A2-X)	Q–Au_101_	—	2.080	2.133
	Si_79_–Au_101_	2.466	2.642	2.645
	C_32_–Zr_100_	2.085	2.085	2.097
	C_34_–Zr_100_	2.090	2.091	2.083
	C_39_–Zr_100_	2.100	2.097	2.093
NO_2__X_Cu_Zr@SiCNT (C1-X)	Q–Cu_101_	—	1.920	1.916
	Si_79_–Cu_101_	2.376	1.966	1.961
	C_32_–Zr_100_	2.084	2.084	2.096
	C_34_–Zr_100_	2.089	2.089	2.080
	C_39_–Zr_100_	2.102	2.099	2.095

a X denotes the n-site and o-site of adsorption. Q denotes the N_102_ and O_104_ atoms present between the surfaces and the NO_2_ gas molecule.

### 3.2 Adsorption study

The most stable adsorption configurations were ensured in the adsorption of NO_2_ gas molecules on the bare and functionalized SiCNT surfaces. To determine the minimum energy configurations, the bare and functionalized surfaces were optimized.^49^ Initially, in a cluster, structural equilibration was carried out using the def2svp basis set. For the best adsorption conformation, two sites of adsorption were considered, namely, the nitrogen and oxygen sites, which were denoted as n-site and o-site, respectively. It is necessary to determine the adsorption energy to know how well an adsorbate is adsorbed by an adsorbent. In this study, the adsorption energy was calculated using the mathematical expression in eqn (1) of the computational details.^50^ Energy calculation was performed for each complex and surface, and then for the NO_2_ gas molecule. Table 2 summarizes the calculated adsorption energy values for all the complexes. The n-site and o-site of adsorption are visualized in Fig. 4. According to Table 2, the adsorption energy values of −2.190 and −2.422 eV were obtained for the Z1-n and Z1-o complexes, respectively. Greater adsorption energies were obtained after functionalizing the surface with transition metals, with the greatest adsorption energies of −3.780 and −2.925 eV corresponding to the C1-o and C1-n complexes, respectively. Similarly, relatively greater energy values were recorded for the A1-n and A1-o complexes, reflecting the adsorption energies of −2.248 and −2.578 eV, respectively. Also, the adsorption energies of −2.512 and −2.265 eV, corresponding to the A2-o and A2-n complexes, respectively, were observed. The o-site of adsorption again exhibits the best adsorption configuration due to the greater adsorption energies recorded. Evidently, the Cu-functionalized surface exhibits the best adsorption potential compared to the Ag- and Au-functionalized Zr@SiCNT surfaces. The basic set superposition error (BSSE) was determined by running BSSE calculations. This was done to correct the adsorption energy calculated from the initial optimization.^51,52^ However, according to this result, it was remarkable that there is no difference between the adsorption energy and the corrected BSSE plus the adsorption energy. This occurrence left the BSSE values at zeros in all the complexes, which was validated by maintaining the decimal places as they appeared during the calculations. Hence, the reliability of the B3LYP-D3(BJ)def2svp computational method and the BSSE method was confirmed.

**Table 2:** The results of the adsorption energy, Fermi energy, work function, fraction of electron transfer, and back donation calculated at the B3LYP-D3(BJ)def2svp level of theory

System	*E*_ad_	*E*_BSSE_ + *E*_ad_	*E*_FL_ (eV)	*Q*_t_ (eV)	Δ*N* (eV)	% Δ*N*	Δ*E* back-donation
NO_2__n_Zr@SiCNT	−2.19016	−2.19016	3.862522	1.06451	−0.00913	−0.91298	−0.9656
NO_2__n_Ag_Zr@SiCNT	−2.24815	−2.24815	3.973817	−0.03452	0.624818	62.48175	−0.3113
NO_2__n_Au_Zr@SiCNT	−2.26472	−2.26472	4.162256	−0.1166	1.196062	119.6062	−1.3731
NO_2__n_Cu_Zr@SiCNT	−2.92501	−2.92501	3.777895	0.17807	0.645692	64.56919	−0.2617
NO_2__o_Zr@SiCNT	−2.42173	−2.42173	3.885788	0.61595	−0.60000	−60.0000	−0.9714
NO_2__o_Ag_Zr@SiCNT	−2.57823	−2.57823	4.112867	0.0417	0.644919	64.49187	−1.3700
NO_2__o_Au_Zr@SiCNT	−2.51232	−2.51232	3.990688	−0.02583	1.773026	177.3026	−0.3113
NO_2__o_Cu_Zr@SiCNT	−3.7801	−3.78010	3.955041	0.20522	0.574286	57.42862	−0.3121

**Fig. 4:** Visualization of the n-site and o-site of adsorption using GaussView.

### 3.3 Electronic property investigation

#### 3.3.1 Energy gap intuition

The concept of energy gap plays a pivotal role in gaining insight into the stability and reactivity of a material. This descriptor is usually determined by employing frontier molecular (FMO) analysis, which primarily and collectively utilizes the highest occupied molecular orbital (HOMO) and the lowest unoccupied molecular orbital (LUMO).^53^ The HOMO and LUMO energies are the fundamental quantities determine the HOMO–LUMO energy gap, and all the other quantum reactivity descriptors are derived.^54^ Koopmans' contributions in deriving these descriptors cannot be overemphasized, given that he established a very important relationship among the descriptors.^55^ Knowledge on the change in the electronic structural properties of a nanomaterial can be acquired by the variation in the energies of the HOMO and LUMO.^56^ Importantly, the difference in energy between the two frontiers molecular orbitals makes it possible to gain useful knowledge on the stability, strength and energy of an adsorbent and the resulting complex after interactions. Upon adsorption, the changes in the electronic structural properties of the NO_2_ gas molecule with the Zr@SiCNT and transition metal-functionalized surfaces were revealed. A thorough literature review showed that an increase in the HOMO–LUMO energy gap is a function of the decrease in the conductivity and increase in the stability of a material.^57^Table 3 shows the HOMO and LUMO energies and the energy gap. Before adsorption, the energy gap values of 2.721, 1.796, 2.422, and 1.333 eV were recorded for the Zr@SiCNT, Ag_Zr@SiCNT, Au_Zr@SiCNT, and Cu_Zr@SiCNT surfaces, respectively. After adsorption, an increase in the energy gap was observed in all cases, where the energy gap values of (3.157, 3.079 eV), (2.721, 2.504 eV), (2.476, 2.667 eV), and (2.504, 2.095 eV) were found for the complexes corresponding to the aforementioned surfaces, respectively, indicating their stability. Considering the site of adsorption, the o-site shows a smaller energy gap compared to n-site of adsorption. This indicates that stability will be better attained when considering the o-site for the adsorption of NO_2_ gas molecules on the surfaces. Also, the lowest energy gap was found for the C1-o complex, reflecting that the o-site of adsorption in the most stable on the Cu-functionalized surface. Also, a relatively smaller energy gap was observed in the other complexes such as A2-n and C1-n, depicting their higher stability compared to the other complexes. Overall, the transition metal-functionalized surfaces show greater stability compared to their non-functionalized counterpart. Fig. 5 shows the HOMO–LUMO plots for the surfaces before adsorption. The HOMO–LUMO plots of the complexes upon n-site and o-site adsorption are presented in Fig. 6.

**Table 3:** HOMO energy (*E*_HOMO_), LUMO energy (*E*_LUMO_), electron potential (EA), ionization potential (IP), electrophilicity index (*ω*), chemical potential (*μ*), chemical softness (*S*), and chemical hardness (*η*), with all units in electron volt (eV) and calculated at the B3LYP-D3(BJ)def2svp level of theory

System	*E*_HOMO_	*E*_LUMO_	*E*_g_	IP	EA	*μ*	*η*	*S*	*ω*
SiCNT	−5.333	−1.878	3.456	5.333	1.878	3.606	1.728	0.289	3.762
Zr@SiCNT	−5.252	−2.531	2.721	5.252	2.531	3.891	1.361	0.367	5.564
Ag_Zr@SiCNT	−4.408	−2.613	1.796	4.408	2.612	3.510	0.898	0.557	6.861
Au_Zr@SiCNT	−5.089	−2.667	2.422	5.089	2.667	3.878	1.211	0.413	6.209
Cu_Zr@SiCNT	−3.946	−2.612	1.333	3.946	2.612	3.279	0.667	0.750	8.064
NO_2__n_Zr@SiCNT (Z1-n)	−5.442	−2.286	3.157	5.442	2.286	3.864	1.578	0.317	4.730
NO_2__n_Ag_Zr@SiCNT (A1-n)	−5.470	−2.748	2.721	5.469	2.748	4.109	1.361	0.367	6.204
NO_2__n_Au_Zr@SiCNT (A2-n)	−5.225	−2.748	2.476	5.225	2.748	3.986	1.238	0.404	6.418
NO_2__n_Cu_Zr@SiCNT (C1-n)	−5.197	−2.694	2.504	5.197	2.694	3.946	1.252	0.399	6.219
NO_2__o_Zr@SiCNT (Z1-o)	−5.425	−2.346	3.079	5.425	2.346	3.886	1.539	0.325	4.904
NO_2__o_Ag_Zr@SiCNT (A1-o)	−5.225	−2.721	2.504	5.225	2.721	3.973	1.252	0.399	6.305
NO_2__o_Au_Zr@SiCNT (A2-o)	−5.497	−2.830	2.667	5.497	2.829	4.163	1.333	0.375	6.499
NO_2__o_Cu_Zr@SiCNT (C1-o)	−4.816	−2.721	2.095	4.816	2.721	3.769	1.048	0.477	6.779

**Fig. 5:** HOMO and LUMO plots for the studied surface prior to adsorption.

**Fig. 6:** HOMO and LUMO plots for the resulting complexes at (a) n-site (b) o-site of adsorption.

#### 3.3.2 Global indices

The chemical quantum descriptors were obtained using the FMO analysis. Based on the generalized Koopmans's hypothesis, the HOMO and LUMO energies have a mathematical relationship, enabling the calculation of the global reactivity indices such as electron potential (EA), ionization potential (IP), electrophilicity index (*ω*), chemical potential (*μ*), chemical softness (*S*), and chemical hardness (*η*).^58,59^ These descriptors as given by the generalized Koopmans' theorem were calculated using the following equations:

2 IP = −*E*_HOMO_

3 EA = −*E*_LUMO_

456

The electrophilicity index (*ω*) was calculated using the following equation:7

The behavior of a material to resist a charged particle in its environment can be understood using chemical hardness.^60^ The related literature on theoretical computations showed that the higher the chemical hardness and chemical potential, the higher the stability and lower the reactivity.^61^ A summary of the global reactivity indices is presented in Table 3. In all cases for the functionalized surfaces, an increase in the chemical potential and hardness values was observed. For example, the values for the Cu-functionalized surface increased from 3.279 eV to 3.946 and 3.769 eV, the values for the Au-functionalized surface increased from 3.986 eV to 3.986 and 4.163 eV, and finally the Ag-functionalized surface showed an increase from 3.510 eV to 4.109 and 3.973 eV, respectively. This increment indicates the higher stability and lower reactivity of the functionalized surfaces. However, the Zr@SiCNT surface, which was not functionalized, showed a decrease in it chemical potential value, thereby indicating its lower stability and higher reactivity. Among the surfaces, the values for the Cu-functionalized surface increased significantly from 0.667 to 1.252 and 1.048 eV for both the n- and o-sites of adsorption, respectively. This again confirmed the inherent stability of the functionalized surfaces, and in particular the Cu-functionalized surface outperformed the studied surfaces due to its relatively large margin. Regarding the site of adsorption, the o-site is the most favorable given that the increment occurred most in the o-site of adsorption. To know whether a chemical species is a strong or weak electrophile, the electrophilicity index (*ω*) is used. Thus, after functionalizing the surface, the *ω* value of 5.564 for the Zr@SiCNT surface increased to 6.861, 6.209, and 8.064 eV for the Ag_Zr@SiCNT, Au_Zr@SiCNT, and Cu_Zr@SiCNT surfaces, respectively, indicating that they are strong electrophiles. Also, due to the relatively higher values observed, the o-site of adsorption is a stronger electrophile than the n-site.

### 3.4 Stabilization energy

As an indispensable approach to gaining useful and reliable knowledge into the pattern of charge transfer within molecules, the natural bond orbital (NBO) analysis, which was developed by Weinhold *et al.*, was employed in this section. To gain further insight into the electronic wavefunction, the localized orbitals such as non-Lewis and anti-bond orbitals were considered. Their applications decipher the knowledge behind the electron density delocalization, re-hybridization, and intra-molecular charge transfer.^62^ The stabilization of the donor–acceptor interactions is due to the exchange of electron densities between the orbitals.

In the present study, we employed the NBO analysis to unravel the pattern of intermolecular delocalization or hyper-conjugation in the adsorption of NO_2_ gas molecules on the bare and functionalized SiCNT surfaces. This analysis enabled us to gain knowledge on the intra and intermolecular interactions in both the donor and acceptor orbitals. Furthermore, the measure of the donor–acceptor interaction stabilization energy, which is called the second-order perturbation energy (*E*^(2)^), leads insights into the type and strength of interaction. Generally, a higher stabilization energy value is associated with strong interactions between electrons and donors and acceptors, indicating a greater degree of conjugation in the system.^63^Table 4 presents the most useful results of the NBO calculation including the second-order perturbation energies, donors and acceptors. According to Table 4, before adsorption, the major charge resonance is that from the anti-bonding charge orbital to the same anti-bonding charge orbital of σ-type (σ* → σ*). However, after adsorption, the major charge delocalization was observed to be the lone pairs to the anti-bonding charge orbital of π-type (LP → π*) in the n-site of adsorption, while in the o-site of adsorption, the charge resonance resulting from the charge transfer from the lone pair to the anti-bonding character of the lone pair (LP → LP*). Additionally, the charge delocalization resulting from charge transfer from the anti-bonding natural orbital between the carbon and zirconium atoms to the same anti-bonding natural orbital between the zirconium and nitrogen atoms (σ*C_34_–Zr_100_ → σ*Zr_100_–N_101_) in the C1-n complex reflects the highest stabilization energy of 1178.00 kcal mol^−1^. The higher energies observed in most cases indicate strong interactions and great stabilization upon adsorption. Therefore, the Cu-functionalized surface exhibits relatively greater stability, and hence easily stabilized compared to its studied counterparts.

**Table 4:** The results of the second-order perturbation-stabilization energy (*E*^(2)^, kcal mol^−1^) calculated at the B3LYP-D3(BJ)def2svp level of theory

System	Donor	Acceptor	*E* ^(2)^/kcal mol^−1^	*E*_(*i*)_ − *E*_(*j*)_	*F*_(*i*,*j*)_
Zr@SiCNT	σ*C_34_–Zr_100_	LP*(3)Zr_100_	561.03	0.03	0.450
Ag_Zr@SiCNT	σ*C_34_–Zr_100_	σ*C_39_–Zr_100_	266.28	0.04	0.422
Au_Zr@SiCNT	σ*C_34_–Zr_100_	σ*C_39_–Zr_100_	646.89	0.02	0.442
Cu_Zr@SiCNT	σ*C_32_–Zr_100_	σ*C_39_–Zr_100_	350.38	0.03	0.429
NO_2__n_Zr@SiCNT (Z1-n)	LP(3)O_104_	π*N_102_–O_103_	128.32	0.22	0.152
NO_2__n_Ag_Zr@SiCNT (A1-n)	LP(3)O_103_	π*N_102_–O_104_	111.03	0.23	0.143
NO_2__n_Au_Zr@SiCNT (A2-n)	LP(3)O_103_	π*N_102_–O_104_	94.59	0.26	0.141
NO_2__n_Cu_Zr@SiCNT (C1-n)	σ*C_34_–Zr_100_	σ*Zr_100_–N_101_	1178.00	0.03	0.602
NO_2__o_Zr@SiCNT (Z1-o)	LP(3)O_104_	LP*(6)Ag_101_	313.70	0.82	0.48
NO_2__o_Ag_Zr@SiCNT (A1-o)	LP(2)O_104_	LP*(6)Au_101_	203.84	0.69	0.371
NO_2__o_Au_Zr@SiCNT (A2-o)	LP*(6)Cu_101_	LP*(6)Cu_101_	140.30	1.03	0.341
NO_2__o_Cu_Zr@SiCNT (C1-o)	LP(3)O_103_	LP*(1)Zr_100_	52.17	1.44	0.350

### 3.5 Visual study of weak interactions

#### 3.5.1 Atoms-in-molecules (AIM) analysis

To gain insight into the intermolecular interaction of a complex system, structural investigations may not be reliable, given that atoms behave in a characteristic way, varying between relatively small regions. In this case, the quantum theory of atoms in molecules (QTAIM), according to Richard F. W. Bader *et al.*, seeks the position of the bonds at the bond critical points to gain insight into the various types of interactions.^64^ The point at which the first derivative of the charge density disappears is known as the critical point,^65^ which makes it possible to identify the position of extrema such as the minima, maxima, and saddle points in the charge density.^66,67^ Specific BCPs localized on the structures visualized in the Multiwfn 3.7 program have a variety of properties, which can be linked to their orientation in space. Moreover, knowledge on hydrogen and non-hydrogen bonding interactions can be gained through the AIM hypothesis.^68^ The topological parameters include electron density, *ρ*(*r*), Laplacian of electron density, ∇^2^*ρ*(*r*), Lagrangian kinetic energy, *G*(*r*), energy density, *H*(*r*), electronic charge density, *V*(*r*), Hamiltonian kinetic energy, *K*(*r*), electron localization function (ELF), (LOL), eigen values *λ*_1_, *λ*_2_, and *λ*_3_, and electrophilicity index of electron density (*ε*). The ratios *G*(*r*)/*V*(*r*) and *λ*_1_/*λ*_3_ were calculated to further probe the nature of the interactions. Table 5 summarizes the results of the topological parameters calculated for before and after adsorption. According to Table 5, the accumulation of electron density between two bonded atoms was observed to have occurred due to ∇^2^*ρ*(*r*) values less than one. It is evident in the literature that the Laplacian of electron density and energy density can be used to determine the nature of interactions. Specifically, classification into non-covalent, partial covalent and strongly covalent can be achieved by simultaneously using the values of ∇^2^*ρ*(*r*) and *H*(*r*). These values follow the order of ∇^2^*ρ*(*r*) > 0 and *H*(*r*) > 0; ∇^2^*ρ*(*r*) > 0 and *H*(*r*) < 0; and ∇^2^*ρ*(*r*) < 0 and *H*(*r*) < 0, corresponding to non-covalent, partial covalent and covalent, respectively. In most cases, the complexes show partial covalent interactions, owing to their values of ∇^2^*ρ*(*r*) > 0 and *H*(*r*) < 0.

**Table 5:** The topological parameters considered at the bond critical points (BCPs) calculated at the DFT/B3LYP/Gen/def2svp/LanL2DZ level of theory

System	Bond	CP	*P*(*r*)	∇^2^*ρ*(*r*)	*G*(*r*)	*V*(*r*)	*H*(*r*)	*G*/|*V*|	ELF	LOL	*λ*_1_	*λ*_2_	*λ*_3_	*λ*_1_/*λ*_3_	*ε*
Zr@SiCNT	C_39_–Zn_100_	147	0.388	−0.188	0.608	−0.471	−0.471	1.291	1.000	0.998	−0.633	−0.617	−0.633	1.026	0.000
	C_31_–Zn_100_	121	0.117	−0.514	0.105	−0.128	−0.128	0.820	0.999	0.998	−0.634	−0.631	−0.634	1.005	−0.249
Ag_Zr@SiCNT	C_46_–Si_88_	99	0.166	−0.427	0.348	−0.106	−0.107	3.283	1.000	0.995	−0.143	−0.142	−0.142	1.007	0.000
	C_49_–S_94_	156	0.109	0.435	0.149	−0.189	−0.399	0.788	0.188	0.324	−0.143	0.715	−0.137	−0.200	0.045
Au_Zr@SiCNT	Si_79_–Au_101_	141	0.703	−0.457	0.244	−0.602	−0.358	0.405	0.665	0.585	−0.501	0.518	−0.474	−0.967	0.057
	C_48_–Si_79_	150	0.108	0.443	0.150	−0.190	−0.396	0.790	0.183	0.321	0.720	−0.134	−0.143	−5.373	0.067
Cu_Zr@SiCNT	Cu_101_–Si_23_	132	0.771	0.262	0.809	−0.962	−0.154	0.841	0.201	0.331	−0.690	−0.594	0.390	1.162	0.161
	C_52_–Si_75_	135	0.109	0.428	0.148	−0.189	−0.412	0.783	0.193	0.328	−0.142	−0.135	0.705	1.052	0.136
NO_2__n_Zr@SiCNT	Zr_100_–O_102_	267	0.475	−0.112	0.335	−0.951	−0.616	0.352	0.860	0.713	−0.117	0.127	−0.122	−0.921	0.043
	Zr_100_–N_101_	261	0.637	0.305	0.786	−0.811	−0.245	0.969	0.121	0.271	−0.824	0.469	−0.821	−1.757	0.004
NO_2__n_Ag_Zr@SiCNT	C_47_–Ag_101_	162	0.911	0.355	0.110	−0.132	−0.215	0.833	0.187	0.325	0.549	−0.918	−0.101	−0.598	0.103
	C_36_–Si_65_	135	0.892	0.441	0.850	−0.595	0.254	1.429	0.165	0.115	0.273	0.215	−0.465	1.270	−1.216
NO_2__n_Au_Zr@SiCNT	C_28_–Au_101_	81	0.166	−0.427	0.348	−0.106	−0.107	3.283	1.000	0.995	−0.142	−0.142	−0.142	1.000	0.000
	C_34_–Zr_100_	107	0.262	−0.937	0.431	−0.320	−0.278	1.347	0.980	0.876	−0.707	0.493	−0.723	−1.434	0.022
NO_2__n_Cu_Zr@SiCNT	C_23_–Cu_101_	34	0.117	−0.515	0.105	−0.129	−0.129	0.814	1.000	0.999	−0.171	−0.172	−0.172	0.994	0.000
	N_102_–Cu_101_	123	0.988	0.476	0.142	−0.166	−0.232	0.855	0.153	0.299	−0.109	0.734	−0.148	−0.149	0.358
NO_2__o_Zr@SiCNT	Zr_100_–N_101_	263	0.308	0.173	0.387	−0.342	0.456	1.132	0.481	0.184	0.113	0.911	−0.309	0.124	−1.339
	Zr_100_–O_102_	262	0.473	0.214	0.517	−0.500	0.169	1.034	0.106	0.256	−0.618	0.331	−0.552	−1.867	0.120
NO_2__o_Ag_Zr@SiCNT	C_23_–Ag_101_	169	0.831	0.205	0.724	−0.937	−0.212	0.773	0.282	0.385	0.364	−0.787	−0.805	−0.463	0.023
	O_104_–Ag_101_	147	0.641	0.315	0.854	−0.921	−0.665	0.927	0.106	0.256	−0.713	0.452	−0.651	−1.577	0.095
NO_2__o_Au_Zr@SiCNT	C_23_–Au_101_	156	0.106	0.241	0.946	−0.130	−0.354	7.277	0.342	0.419	0.447	−0.100	−0.105	−4.47	0.050
	Si_76_–O_103_	105	0.105	0.151	0.946	−0.151	−0.570	6.265	0.335	0.415	−0.133	0.421	−0.137	−0.316	0.026
NO_2__o_Cu_Zr@SiCNT	Si_79_–Cu_101_	132	0.105	0.355	0.115	−0.142	−0.268	0.810	0.249	0.365	0.590	−0.114	−0.121	−5.175	0.056
	Si_76_–O_103_	169	0.101	0.372	0.130	−0.166	−0.366	0.783	0.191	0.327	−0.127	−0.124	0.624	1.024	0.022

The results obtained can be further confirmed using the values of the ratio of *λ*_1_/*λ*_3_. Similar to that reported in ref. 69, the values of *λ*_1_/*λ*_3_ were observed to be less than one in the case of the C1-n complex with *λ*_1_/*λ*_3_ values of 0.994 and −0.149 for the C_23_–Cu_101_ and N_102_–Cu_101_ bonds, respectively, indicating the presence of strong intermolecular interactions. Similarly, a small *λ*_1_/*λ*_3_ value of −5.175 was calculated for the Si_79_–Cu_101_ bond, which is less than one, indicating the presence of intermolecular interactions. Furthermore, to confirm the results of the characteristic interactions, the *G*/|*V*| ratio was utilized. The nature of interactions is classed as covalent, partial covalent, and non-covalent when the *G*/|*V*| ratios are greater 1, between 1 and 0.5, and less than 0.5, respectively.^70,71^ Again, the partial covalent type of interaction was confirmed by the calculated *G*/|*V*| ratio values of between 1 and 0.5 in most cases. Insight into the stability of bonds and the regions of charge density accumulation can be gained using the ellipticity of electron density (*ε*).^72^ A stable interaction is depicted by a small bond ellipticity value (*ε* < 1) at the bond critical points. Small *ε* values less than unity were found for the C1-o complex (0.056, 0.022) and C1-n complex (0.000 and 0.358), depicting the stability of the Cu-functionalized surface in both sites of adsorption, respectively. In all cases, as shown in Table 5, the ellipticity values are less than one, suggesting the stability of the surfaces.

#### 3.5.2 RDG analysis

The notion of non-covalent interactions in real space can be understood using the electron density and its derivatives.^73^ Using the 3D iso-surface, the reduced density gradient (RDG) analysis makes it possible to gain insight into the weak interactions present in complexes.^74^ The previous sections showed that the studied complexes exhibit weak interactions; however, here knowledge on the weak interactions was obtained based on van der Waals forces, π effect, hydrophobic effects, and electrostatic attractions. All the computational calculations were carried out using the Multiwfn program, which in the same spatial range, produces grid data with high quality. Knowledge of the degree of interactions as well as the type of bond was obtained *via* the RDG clusters, *λ*_2_, and reduced density gradient spikes. The product of the electron density, *ρ*(sign(*λ*_2_)*ρ*), with the second eigen value of the Hessian matrix (*λ*_2_) is the fundamental working principle of the RDG plot.^75^ The interactions are often shown by an isosurface with color fills. As depicted in the 3D iso-surface plots, the green color implies van der Waals force of interaction and suggests low electron density, whereas the deep-blue iso-surface indicates the presence of significant forces of attraction. Fig. 7 shows the NCI 3D iso-surface plots. The presence of non-directional attraction as a result of van der Waals dispersion forces was observed due to the green iso-surfaces dominating the interatomic spaces. Therefore, the nature of closed-shell forces were ascertained over the region of the RDG surface.

**Fig. 7:** 3D iso-surface plots for the complexes in both n-site and o-site of adsorption.

### 3.6 Density of states (DOS) analysis

The description of the energy difference between the highest occupied orbital (HOMO) and the lowest unoccupied molecular orbital (LUMO) of a complex, using the Fermi energy level, TDOS and PDOS peaks can be done in the context of density of states (DOS) analysis.^76^ The changes that occur due to interactions between the NO_2_ gas molecule and the surfaces can be visualized using DOS. Insight into the electronic pattern and the most permissible energy for the HOMO to LUMO transition as a result of interactions can be gained using the DOS plots.^77^ Upon adsorption, the changes in electronic properties of the adsorbent materials can be understood from the total density of states (TDOS). The changes in the conductivity of a material can be shown by the shift in the TDOS peaks and changes in their intensity. The Multiwfn function analyser 3.7 and Origin software package were used to plot the DOS for the nano-surfaces after adsorption, as shown in Fig. 8. It can be seen from the plot in Fig. 8 that the functionalization of the surface leads to an increase in the electronic state near the Fermi energy level. The drop around the Fermi energy level after adsorption suggests an increase in conductivity and sensitivity of the surfaces to NO_2_ gas.^78^ The morphology of the functionalized surfaces and the non-overlapping area are the reasons for the similarity in their DOS plots. The wide region of the DOS near the Fermi energy level is an indication that there are more electrons in the HOMO that are readily available to conduct energy upon their transition. Furthermore, higher conductivity was observed for the transition metal-functionalized surfaces, which can be attributed to the high Fermi energy level computed. Thus, the functionalized surfaces have an advantage over the bare Zr@SiCNT surface. Lastly, the individual contribution of the atomic orbitals of the complexes results in the total density of states (TDOS) and the partial density of state (PDOS) in the plot. Due to the unfavorable overlapping within the orbital phase, the anti-bonding characteristics are shown using the overlap partial density of states (OPDOS).

**Fig. 8:** DOS plots showing the TDOS, PDOS, and OPDOS for the studied complexes.

### 3.7 Molecular dynamic simulations

The structural, dynamical and thermodynamic behaviors of the studied systems were further studied using molecular dynamic (MD) simulations. Information on how the NO_2_ molecule approaches, engages, and adheres to the surface of the bare and TM-functionalized zirconium-doped silicon carbide nanotubes (Zr@SiCNT) was obtained using MD simulations.^79,80^ Given that metal dopants have a strong influence on the sensing properties of surfaces, structural modifications using these dopants becomes a key part in deigning materials with enhanced functionalities. Hence, MD simulations were performed to gain further insight into how enhanced adsorption potential and stability of these materials can be attained through structural modifications. Briefly, MD simulations were performed to determine the optimal NO_2_ detection attributes. The results of the simulation calculations such as total, potential, and kinetic energies are presented in Tables S1–S3 of the ESI,† corresponding to the surfaces, n-site, and o-site of adsorption, respectively. It can be observed that upon adsorption, the total energy and potential energy values increase (see Tables S1–S3†). According to Table S2,† the initial total energies of 288.863, 361.520, 222.790, and 187.956 kcal mol^−1^ were determined for the Z1-n, A1-n, A2-n, and C1-n complexes in the n-site of adsorption, respectively. Similarly, for the o-site of adsorption, the Z1-o, A1-o, A2-o, and C1-o complexes reflect the initial total energy corresponding to 146.233, 305.996, 213.363, and 329.161 kcal mol^−1^. Furthermore, the initial potential energy values were 199.146, 270.915, 132.186 and 97.351 kcal mol^−1^ for the Z1-n, A1-n, A2-n, and C1-n complexes, respectively. However, upon simulation, the potential energy increased, where the Z1-n, A1-n, A2-n, and C1-n complexes exhibited values of 241.591, 316.830, 163.826, and 143.941 kcal mol^−1^, respectively (see Table S1†). Similarly, as observed for the o-site of adsorption, the potential energy increased from the initial values of 56.516, 215.391, 122.758, and 238.556 kcal mol^−1^ for the Z1-o, A1-o, A2-o, and C1-o complexes to the final values of 102.623, 264.480, 163.526, and 280.427 kcal mol^−1^, respectively. Due to the above-mentioned adjustment from initial to final values for the potential energy, a favorable interaction is considered to have occurred between the NO_2_ gas and the labelled surfaces. Initially, the kinetic energy values were found to be as follows: Z1-n complex: 89.716 kcal mol^−1^; A1-n complex: 90.605 kcal mol^−1^; A2-n complex: 90.605 kcal mol^−1^; and C1-n complex: 90.605 kcal mol^−1^. Alternatively, in the final stage of simulation, the kinetic energy decreased in value to the final value, as follows: Z1-n complex: 47.656 kcal mol^−1^A1-n complex: 44.959 kcal mol^−1^. Similarly, a decrease to 59.131 and 44.342 kcal mol^−1^ was observed for the A2-n, and C1-n complexes, respectively. At the o-site of adsorption, a consistent decrease from the initial to final value was observed, where the Z1-o, A1-o, A2-o, and C1-o complexes showed a decrease in kinetic energy values from 89.716, 90.605, 90.605, and 90.605 kcal mol^−1^ to 43.978, 42.037, 50.332, and 49.098 kcal mol^−1^, respectively (see Table S3†). These variations, as observed during the simulations, can used in the design of new surfaces that are suitable for the fabrication of sensors and drug carriers. These changes can be related to the molecular motion, where a decrease in kinetic energy leads to a decrease in the molecular motion of the system. Fig. 9 shows the dynamic temperature fluctuation for the studied surfaces.

**Fig. 9:** Dynamic fluctuation in temperature for the labelled surfaces.

The visualization of the fluctuation in dynamic temperature for the adsorption of NO_2_ gas molecules on the nanotubes is presented in Fig. 10 and 11. The temperature for all the systems was initially recorded as 298 K, with a consistent decrease across all the resulting complexes. In the case of the Z1-n, A1-n, A2-n, and C1-n complexes, a decrease to 158.294, 147.872, 194.483, and 145.840 K, respectively, was confirmed in the n-site of adsorption. Similarly, a consistent decrease was observed for the Z1-o, A1-o, A2-o, and C1-o complexes, where their temperature decreased to 146.078, 138.261, 165.543, and 161.485 K, respectively. These results reveal the thermodynamic characteristics and stability of the studied nanotubes. The mean square displacement (MSD) was employed to determine the bond strength and restoring forces of the nanotubes, wherein high restoring forces are associated with a low MSD, and then decrease in atomic mobility.^81^ Additionally, a strong and firm bond are attributes of a lower MSD and atom mobility. The small MSD values observed across the systems indicate that the adsorption of NO_2_ gas will force the structure to deform over time. In summary, the inter-atomic interaction results in a fluctuation in temperature, which indicates the presence of thermal energy.

**Fig. 10:** Dynamic fluctuation in temperature for the adsorption of NO_2_ gas molecule on the nanotube at n-site of adsorption.

**Fig. 11:** Dynamic fluctuation in temperature for the adsorption of NO_2_ gas molecule on the nanotube at the o-site of adsorption.

### 3.8 Sensor mechanisms

Here, the parameters that determine the effectiveness of sensor materials are discussed. These parameters are known as sensor parameters or sensor mechanisms. One of the essential parts of developing a sensor device is the knowledge of materials with the potential to sense or detect the targeted adsorbate. Owing to this reason, this section further aims to substantiate and solidify the insights gained on the studied surfaces in the previous sections using the sensor parameters such as charge transfer (*Q*_t_), Fermi level (*E*_FL_), electrical conductivity (*σ*), fraction of electron transfer, back donation, and sensor reusability, which is usually measured using the recovery time.

#### 3.8.1 Charge transfer mechanism

The charge transfer mechanism can be determined based on the chemical quantum descriptors, which are all dependent on the HOMO and LUMO energies. Based on the distribution of electron density in the studied systems, it was possible to study the charge transfer mechanism. Therefore, partitioning the electron density into individual atoms or molecular fragments was possible using this approach. Considering the charges of each bare and functionalized SiCNT surface before and after the adsorption of NO_2_ gas molecules, the charge transfer was calculated using eqn (8), as follows:

8 *Q*_t_ = *Q*_adsorption_ − *Q*_isolated_

where *Q*_t_ denotes the charge transfer and *Q*_isolated_ and *Q*_adsorption_ are the charge transfer before and after adsorption, respectively. According to the literature, a negative *Q*_t_ value indicates the transfer of electrons from the adsorbate to the adsorbent material, whereas a positive value suggests electron transfer from the adsorbent material to the adsorbate.^82^ Unlike the Hirshfeld analysis used in the study of charge transfer, the Bader charge analysis is adopted in this section due to the sensing nature this work. Also, the charge transfer can be analyzed using the HOMO and LUMO orbitals, with the HOMO–LUMO energy gap used as a key parameter. Table 2 shows the results of the charge transfer (*Q*_t_) in the o-site and n-site of adsorption for the complexes. The computed results were found to be significant due to the positive *Q*_t_ values obtained in most cases. Also, according to the literature, a positive *Q*_t_ value is often associated with good sensor behavior for a material, depicting that charge transfer from the adsorbent to the adsorbate shows some level of consistency. A higher charge transfer (*Q*_t_) value reflects obvious charge flow between the studied surfaces and the NO_2_ gas molecule. Adsorption on the Zr@SiCNT surface reflects the greatest charge transfer of 1.065 and 0.616 eV in both the n-site and o-site of adsorption, respectively, suggesting that a substantial amount of charge must have been transferred between the adsorbent and the adsorbate. Similarly, the Cu-functionalized Zr@SiCNT surface possesses the highest charge transfer in both the n-site and o-site of adsorption, with *Q*_t_ values of 0.178 eV and 0.205 eV, respectively. However, the negative charge transfer values observed for adsorption on the Ag_Zr@SiCNT (*Q*_t_ = −0.035 eV) and Au_Zr@SiCNT (*Q*_t_ = −0.117 eV) surfaces indicate a negative influence on the sensor behavior of these materials. Thus, the o-site of adsorption can be considered the best adsorption site, owing to its positive charge transfer values. Given that this result agrees with that obtained in the previous sections from the adsorption study, energy gap, and other sensor mechanisms, Cu-functionalized Zr@SiCNT surface reflects the highest sensitivity among the studied surfaces.

#### 3.8.2 Fraction of electron transfer (FET) and back donation

As demonstrated in Section 3.3, the chemical quantum descriptors of electronegativity and global hardness are indicators of the electron transfer in the nanotubes, thereby denoting the required amount of energy to spark a change in the electron density of any system. A lower propensity for charge transfer between an adsorbate and adsorbent is often due to the high energy barrier for electron transfer.^83^ This scenario can be linked to the FET, where a lower global hardness leads to a higher FET, indicating an increase in electron transfer upon adsorption.^84^ In the case of a higher FET value, the influence of electronegativity on the likelihood of electron transfer from the bare and functionalized SiCNT surfaces is the pathway to gaining insight into the direction and strength of charge transfer. In the adsorption process, the FET values show the level of electron transfer between the adsorbent and adsorbate. The electron transfer is widely applied in field-effect transistor and chemiresistive sensors as a gas sensing mechanism.^85^

The portion or part of electrons that are transferred from the adsorbent to the adsorbate as a result of the adsorption process can be quantified by the FET values. Also, the extent of electron donation from a gas molecule to the adsorbent material is known as back donation. In fact, the relationship between the FET and back donation is that back donation is the reverse process of FET, which is the transfer of electrons back from the gas molecule to the surface. Gómez and team shed light on how the contact between the NO_2_ gas molecule and bare and functionalized SiCNT surfaces may be controlled by an electrical back-donation mechanism.^86^ The fraction of electron transferred (Δ*N*) and its back donation was computed based on the Pearson theory. The fraction of electron transferred (Δ*N*) is calculated using eqn (9), as follows:9where *χ* and *η* denote the electronegativity and chemical hardness value, respectively. Also, the back donation (Δ*E*) was calculated using eqn (10), as follows:10

In a sensor material, back-donation is considered good when *η* > 0 and Δ*E*_Back-donation_ < 0. Based on the contact with the surface, the stability can be compared given that it increases with an increase in the chemical hardness of the system. A higher FET value reflects the transfer of electrons from the adsorbent to the adsorbate, resulting in strong adsorption, with an increase in the adsorption potential. Similarly, a higher back donation value suggests good electron donation from the NO_2_ gas molecule back to the SiCNT surfaces, thereby making the complex stable. The calculated FET (Δ*N*) and Δ*E*_Back-donation_ values are summarized in Table 2. According to Table 2, all the complexes reflect relatively high Δ*E*_Back-donation_ values. The Δ*E*_Back-donation_ value of −0.262 eV was observed for adsorption on Cu_Zr@SiCNT in the n-site of adsorption. Similarly, the Cu-functionalized Zr@SiCNT surface has a Δ*E* value of −0.312 eV in the o-site of adsorption. According to Table 2, all the studied complexes exhibit high FET values. The FET values of 64.569 and 57.429 eV were recorded for the C1-n and C1-o complexes, respectively, suggesting efficient electron transfer from the nanotube to the NO_2_ gas molecule and strong adsorption and enhanced adsorption capacity.

#### 3.8.3 Electrical conductivity

The concept of electrical conductivity involves the flow of current through the adsorbent material under an electric field. In the case of sensors for gas, the concentration of gas molecules can be determined based on the change in electrical conductivity. This also enables the movement of electrons from the valence band to the conduction band.^87^ The inverse relationship between the electrical conductivity and energy gap can be illustrated using eqn (11), as follows:

11 *σ* = *AT*^2/3^e^(*E*_g_/2*KT*)^

where *σ*, *A*, *T* and *K* denote the electrical conductivity, constant, temperature, and Boltzmann constant, respectively. According to Table 2 and eqn (11), it is evident that an increase in conductivity leads to a decrease in the energy gap, following the order of Z1-o (3.079 eV) > A2-o (2.667 eV) > A1-o (2.504 eV) > C1-o (2.095 eV), with the Cu-functionalized surface showing the most conducting surface. Hence, it exhibits the most potential as an NO_2_ gas sensor material.

#### 3.8.4 The reusability of the sensor material

The ability of a sensor material to be reused has become indispensable when designing a sensor device. It is worthwhile to note that the time it takes for an adsorbent material to desorb an adsorbate that it initially adsorbed is known as the recovery time. Based on a literature review, a shorter recovery time is often required for a good sensor device.^88^ This is because the quick recovery of a pollutant from sensor devices ascertains the reusability of their materials. Based on the conventional transition-state theory, the recovery time can be calculated using eqn (12), as follows:

12 *τ* = *V*_0_^−1^e^−*E*_ad_/*KT*^

where *V*_0_ denotes the attempt frequency, which is (10^12^ s^−1^) and *K* denotes the Boltzmann constant and is approximately equal to 8.62 × 10^−5^ eV K^−1^. Table 6 presents the recovery time of the investigated materials calculated using eqn (12). The higher the magnitude of the negative adsorption energy, the longer the recovery time. However, in the present work, the recovery time will not be prolonged given that the adsorption energy values obtained fall in the small range of −2.19016 to −3.7801 eV, which are moderate. The results obtained here are in excellent accordance with other theoretical reports.^89^

**Table 6:** The result of the recovery time calculated at the B3LYP-D3(BJ)def2svp level of theory

System	*E*_ad_ (eV)	τ (s)
NO_2__n_Zr@SiCNT (Z1-n)	−2.19016	2.6227 × 10^28^
NO_2__n_Ag_Zr@SiCNT (A1-n)	−2.24815	3.0827 × 10^29^
NO_2__n_Au_Zr@SiCNT (A2-n)	−2.26472	6.2335 × 10^28^
NO_2__n_Cu_Zr@SiCNT (C1-n)	−2.92501	9.554 × 10^41^
NO_2__o_Zr@SiCNT (Z1-o)	−2.42173	4.9238 × 10^32^
NO_2__o_Ag_Zr@SiCNT (A1-o)	−2.57823	3.806 × 10^35^
NO_2__o_Au_Zr@SiCNT (A2-o)	−2.51232	2.3127 × 10^34^
NO_2__o_Cu_Zr@SiCNT (C1-o)	−3.7801	5.7626 × 10^57^

### 3.9 Comparative study on previous adsorption of NO_2_ gas pollutant

This section focuses on the properties of a state-of-the-art NO_2_ detecting material to show how much the Cu-functionalized SiCNT outperforms the state-of-the-art material. Related theoretical literature was gathered, analyzed, and compared to the present work. In most cases, the Cu-functionalized SiCNT outperforms the state-of-the-art material (see Table 7).

**Table 7:** Comparison between previous studies on NO_2_ gas pollutant adsorption and the present work

Previous studies on NO_2_ gas adsorption	Ref.
Title: A first-principle investigation of NO_2_ adsorption behavior on Co, Rh, and Ir-embedded graphitic carbon nitride: looking for highly sensitive gas sensor	90
There are cases where the adsorption energy was moderate (−0.231, −2.63, and −1.69 eV for pristine/NO_2_, Co/NO_2_, and Rh/NO_2_, respectively); however, the large negative adsorption energy of −4.47 eV for the Ir/NO_2_ complex, with the recovery time of 3.94 × 10^63^ s will prolong the recovery of the NO_2_ gas pollutant, thereby affecting the reusability of device	
Title: Adsorption of CO, NH_3_, NO, and NO_2_ on pristine and defective g-GaN: improved gas sensing and functionalization	91
The adsorption energy of −0.364 eV was obtained for NO_2_ gas on the pristine g-GaN surface. However, the adsorption energy was enhanced when the NO_2_ gas was absorbed on defective g-GaN surface. Due to the aforementioned small energy, the present work has a relatively higher adsorption as compared to this, showing that Cu-functionalized SiCNT outperforms the studied pristine and defective g-GaN surfaces	
Title: Enhancing the sensing performance of zigzag graphene nanoribbon to detect NO, NO_2_, and NH_3_ gases	92
Upon NO_2_ gas adsorption on ZGNR, ZGNR–O, ZGNR–OH, and ZGNR–O–OH, the adsorption energy obtained was −0.225, −0.212, −0.618, and −0.953 eV respectively. However, although the adsorption was improved *via* functionalization with small molecules, it was lower than that obtained in the present work. The Cu-functionalized SiCNT surface shows stronger adsorption towards NO_2_	
Title: Selective adsorption function of B_16_C_16_ nano-cage for H_2_O, CO, CH_4_ and NO_2_	93
NO_2_@B_16_C_16_ complex does not only reflect a very high adsorption energy of −16.6 eV, indicating very strong adsorption, but also exhibits the highest energy gap of 3.69 eV. This does not correlate with the mechanistic property of a sensor material, according to its lowest conductivity among the studied systems. Besides, the NO_2_ gas will be prolonged by over four-times than that on the Cu-functionalized SiCNT surface during recovery. Hence, the Cu-functionalized SiCNT surface exhibits a better sensing performance	

## 4 Conclusions

The adsorption of NO_2_ gas molecules on bare and transition metal-functionalized SiCNT surfaces was investigated using density functional theory (DFT) computation at the B3LYP-D3(BJ)def2svp level of theory. To determine the best adsorption configurations, different sites of adsorption were considered, wherein the n-site and o-site of adsorption were used. Insights into the sensing attributes of the bare and transition metal-functionalized SiCNT surfaces were gained through electronic descriptors such as the FMO and NBO analyses; the study of weak interactions such as QTAIM and RDG analyses; the knowledge of the electronic pattern *via* TDOS and PDOS peaks, DOS analysis; and sensor mechanisms to ascertain the results obtained from these investigations. Herein, the following conclusions were drawn:

(1) Due to adsorption, the morphology of the nanotubes are altered, as seen from the shortened and elongated bond lengths.

(2) The adsorption phenomenon is best described as chemisorption, owing to the negative adsorption enthalpy. The Cu-functionalized surface reflects the greatest adsorption energies of −3.780 and −2.925 eV, corresponding to the o-site and n-site of adsorption, respectively, which implies that the Cu-functionalized surface is the best at adsorbing NO_2_ gas among the studied surfaces.

(3) The C1-o complex exhibits the lowest energy gap of 2.095 eV, indicating that the Cu-functionalized surface is the most stable at the o-site of adsorption. Also, a relatively smaller energy gap was observed in the other complexes such as A2-n and C1-n, depicting their stability compared to the other surfaces.

(4) In most cases, partial covalent interactions were observed, except when strong and non-covalent interactions were recorded. The stability of the Cu-functionalized surface in both sites of adsorption was due to the small ellipticity (*ε*) values found in the C1-o complex (0.056, 0.022) and C1-n complex (0.000 and 0.358), respectively.

(5) The green colour of the 3D RDG maps indicates that all the complexes have low van der Waals interactions.

(6) The sensor mechanisms confirmed that the Cu-functionalized surface exhibits the best sensing attribute, through its superior sensitivity, conductivity, and enhanced adsorption capacity.

## Ethical statement

We want to clarify that our research did not require ethical approval, and we have accordingly updated the statement to reflect this information.

## Data availability

All information regarding to this study are presented in this document and the ESI.†

## Author contributions

Ismail O. Amodu: investigation, methodology, supervision. Faith O. Akor: writing, analysis and manuscript first draft: Innocent Benjamin and Oluwatobi A. Olaiya: visualization, analysis and writing. Miracle N. Ogbogu: analysis, reviewing, writing, and editing. Adedapo S. Adeyinka: resources and software, Hitler Louis: project conceptualization, design, resources and supervision.

## Conflicts of interest

All authors declare zero financial or inter-personal conflict of interest that could have influenced the research work or results reported in this research paper.

## Supplementary Material

RA-014-D3RA08796D-s001
